The article "Bioinformatics Method Was Used to Analyze the Highly Expressed Gene FAM83A of Breast Cancer in Young Women" was retracted in 2023. Reasons: signs of a paper mill; compromised peer review; unreliable results or conclusions.

# Bioinformatics Method Was Used to Analyze the Highly Expressed Gene FAM83A of Breast Cancer in Young Women

**DOI:** 10.1155/2022/5358030

**Published:** 2022-03-29

**Authors:** Yongzhe Tang, Hao Wang, Qi He, Yuanyuan Chen, Jie Wang

**Affiliations:** ^1^The International Peace Maternal and Child Health Hospital, School of Medicine, Shanghai Jiao Tong University, Shanghai, China; ^2^Shanghai Key Laboratory of Embryo Original Diseases, Shanghai, China; ^3^Teaching Center of Experimental Medicine, Shanghai Medical College, Fudan University, 138 Yixueyuan Rd, Shanghai 200032, China

## Abstract

**Objectives:**

Preliminary analysis of breast cancer related to unknown functional gene FAM83A through bioinformatics knowledge to inform further experimental studies. Select high expression genes for breast cancer and use bioinformatics methods to predict the biological function of FAM83A.

**Methods:**

Genes with significant differences in expression between breast tumors and normal breast tissue libraries were selected from CGAP's SAGE Digital Gene Expression Displayer (DGED) database. An unknown functional gene, FAM83A, which is highly expressed in breast cancer, was screened. We performed an analysis of the gene structure, subcellular localization, physicochemical properties of the encoding products, functional sites, protein structure, and functional domains.

**Results:**

Through SAGE DGED, a total of 185 genes with expression differences were found. The structure and function of FAM83A have ideal predictions, and it is generally determined that this gene encodes a nuclear protein with a nucleoprotein. The active site of PLDc and the functional domain of DUF1669 can be involved in signal transduction and gene expression regulation in tumorigenesis and metastasis. Digital gene representation of the Tumor Genome Project Data Library was used to select differentially expressed genes in breast cancer tissue and breast benign tumor tissue.

**Conclusion:**

Studies show that FAM83A is a potential research target associated with tumorigenesis and metastasis. Initial tests confirmed the expression of this gene. Lay a solid foundation for further research learning. FAM83A is a highly expressed gene in breast cancer and can serve as a target for studying molecular mechanisms in breast cancer.

## 1. Introduction

FAM83A, the family member A gene with a sequence similarity of 83, is a protein-coding gene with a domain whose function needs to be defined. It is the earliest identified recessive tumor gene, which is upregulated in lung cancer, liver cancer, breast cancer, and other malignant tumors, promoting cancer cell proliferation, migration, invasion, and mesenchymal transformation of epithelial cells [1]. Current research recognizes a variety of microRNAs as tumor suppressor genes, with circRNA or long noncoding RNA on top of them Swim, directly or indirectly targeting. FAM83A forms an axis acting on signaling pathways, restraining the emergence and exacerbation of cancer, but detailed molecular mechanisms stay ahead. This article reviews the expression and role of FAM83A in breast cancer [2].

Malignancies originate from abnormal cell division and proliferation. The FAM83 family genes are extensively involved in this process. Many of their family are oncogenes, with significantly increased expression levels in the tumors. FAM83A is a family member A gene with a sequence similarity of 83, also known as BJ-TSA-9. It is located on chromosome 8q24 and is a protein-coding gene. It contains a domain whose function requires a 1669 definition and was identified as a recessive tumor gene. Studies has demonstrated that FAM83A has a high expression capacity in malignancies such as lung cancer, liver cancer, and pancreatic cancer and is associated with tumor proliferation, metastasis, invasion, drug resistance, and epithelial stromal transformation. Thus, FAM83A is closely associated with malignancy [3].

Malignant tumors are serious diseases that endanger human health, and the mortality rate of malignant tumors in China has shown a clear upward trend. In developed countries, breast cancer is the number one cancer in women. The incidence of breast cancer in China is showing a trend of younger age [4].

Breast cancer is a serious threat to women's physical health, and the incidence rate has jumped to the top of the incidence of cancer among women in China. X-ray screening is limited by imaging, leaving many patients without the opportunity for initial discovery. Screening for tumor biomarkers has important implications for the early detection of breast cancer and has become the main focus of current research. With the rapid growth of biological data and rapid advances in computer technology, emerging disciplines such as bioinformatics have developed at an unprecedented rate, especially in bioinformatics [5]. Many biological signs of the disease have now been identified. This paper uses the Tumor Genome Anatomy Project (CGAP) Gene Expression Analysis (SAGE) database to provide an overview of the gene expression profile of tumor tissues and select new breast cancers. The role of highly expressed genes and functionally ambiguous FAM83A in tumor production is being mined. The biological function of this gene lays the foundation for its molecular mechanism of involvement in the development of breast cancer [6].

Breast cancer is the most prevalent malignant tumor in female. It is an important reason for the death of global female sex cancer. In the global field, there were roughly 2.1 million newly diagnosed female breast cancer cases in 2018, accounting for nearly a quarter of female sexual cancer cases. With changes in screening procedures and treatment procedures, the survival rate of breast cancer patients has increased. The survival time of different patients with breast cancer is significantly different. The study reported that 5-year stage survival in stage 1 breast cancer is nearly 100%, and these patients diagnosed with stage IV breast cancer has decreased to 26%, suggesting lower survival in the number of advanced diseases in breast cancer [7]. Traditional treatment modalities, such as surgery, chemotherapy, and radiotherapy, do not provide better therapeutic results for patients with advanced breast cancer. The heterogeneity of breast cancer tumors makes the therapeutic effect of breast cancer different from individual to individual. The pathogenesis of breast cancer is complex, and its hidden molecular mechanisms are not yet fully understood. Therefore, there is an urgent need to explore more transcendent and economical biological markers to anticipate the prognosis of breast cancer, to open up better treatment methods, and to better understand the targets of its hidden organs [8].

Breast cancer is one of the most common malignant tumors, that is, the highest incidence of malignant disease among female tumors. Breast cancer can be divided into 4 subtypes (luminal A, luminal B, HER2, and triple negative breast cancer), following the indications of the estrogen receptor (ER), progesterone receptor (PR), and human epidermal growth factor receptor-2 (HER2). Individualized treatments that follow the biological characteristics of differential breast cancer subtypes and clinical pathological staging of responses can achieve a 5-year survival rate of more than 90% for breast cancer [9]. However, the recurrence and transfer of breast cancer is still a difficult problem. In addition, some breast cancer subtypes, such as triple-negative breast cancer, have always been a difficult point in clinical treatment because of the lack of effective therapeutic targets. Therefore, identifying the important genetic pathways corresponding to the changes in breast cancer is conducive to understanding the potential pathogenesis of breast cancer, or it will provide reference for clinical treatment to explore more confirmed and therapeutic targets [10].

Since the advent of gene chip technology and high constant sequencing skills, bioinformatics has changed rapidly, and many biotechnical markers of diseases have now been discovered. From well-informed public databases such as the Gene Expression Omnibus (GEO) and the TCGA (The Cancer Genome Atlas) Value Library, the gene sequencing data can be obtained. Using the bioinformatics step, the gene indication values in the numerical database are clustered, summarized, explained, and visualized [11]. The efficacy of genes and the function of genes can be predicted, the pathogenesis at the genetic level of the disease can be understood, and the recessive biological targets can be perceived. Therefore, it is the theoretical basis for the development of targeted medicinal materials for the molecules of the disease and the supply of precise healing. This study combines breast cancer gene indication values with clinical survival elaboration to select important genes and important information pathways; given that genes selected during survival are probably more clinical, they may provide new ideas for breast cancer consultation and treatment [12]. In recent years, in view of the fact that microarrays of high-throughput platforms have been transformed into genetic or epigenetic transformations that are the focus of the cancer discovery process and the prospective organisms of cancer consultation and prognosis. Effective materials for landmarks. In bioinformatics elaboration in view of the gene chip, the selection of data, the total elaboration, the visualization of the wrist, and the molecular interaction network will be explained and other steps to integrate massive and chaotic biotechnological information, explore hidden biological markers, and provide new strategies for the treatment of diseases [13].

Due to the characteristics of high morbidity and high mortality, many scholars attended breast cancer seminars. Initial consultation and molecular targeted therapy necessitate affirmative changes in the key genes of breast cancer progression, conversion, and poor prognosis. The manifestations of VEGF and FAM83A correspond significantly to the various clinical pathological characteristics and prognosis of breast cancer patients and can be regarded as the therapeutic target of breast cancer [14]. Studies in the literature suggest that some molecular markers are associated with poor prognosis in breast cancer; for example, the human-encoded FAM83A gene is highly expressed in breast cancer. This study was aimed at exploring the important differential factors in the Gene Expression Omnibus (GEO) gene indication database, hoping to obtain more biological information corresponding to the prognosis of breast cancer and provide new targets for the treatment of breast cancer [15].

## 2. Materials and Methods

### 2.1. Data Acquisition

In order to obtain the gene expression value set of breast cancer, this study downloaded three breast cancer value sets (http://www.ncbi.nlm.nih.gov/geo/) from the GEO database, namely, GSE54002, GSE29431, and GSE61304, all of which are based on the GPL570 level platform. GSE54002 includes 417 breast cancer samples and 16 common samples. GSE29431 included 54 breast cancer samples and 12 common samples: 15 of the 54 breast cancer samples were HER2 immune to histochemical division into 3+ and accompanied by HER2 gene amplification; 26 cases were scored 2+, of which 13 cases were accompanied by HER2 gene amplification and 13 cases were not accompanied by HER2 gene amplification; 13 cases were divided into 0/1+ and were not accompanied by HER2 gene amplification [16]. GSE61304 included 58 breast cancer samples and 4 common samples: 18 of the 58 breast cancer samples were ER+PR+, 19 were ER-PR-, 4 were ER+PR-, 1 was ER-PR+, and the remaining 16 samples were not elucidated. Conduct chip batch correction through NCBI's own tools. The differences in expression represented by breast cancer and pool 2 types of tags (short tags and long tags) of selected people are of significance (F2≥, *p* ≤ 0.05) gene 185. After reviewing the data to exclude genes with known function, a new gene with unknown function FAM83A was selected from 52 genes with high expression in breast cancer (FAM83A in the short tag library). The ratio of expression in breast cancer to normal breast tissue is 14.09. In the long tag library, this ratio is 3.68 [17].

### 2.2. Screening for Differentially Expressed Genes

Upload and download the software on the Bioconductor website in RStudio software (text 3.4.0). Pack to illustrate the 3 breast cancer numerical sets described above. The first application of affy package into the CEL archive, the application of simpleaffy package to evaluate the quality of microarray data, and the RMA calculation method in the gcrma package presolved the initial value. The gene filter package was used to screen non-super-absolute joint probes and probes with low numerical quality, and limma package was used to hold a total of differential gene indications of the total academic study. Gene expression changes multiple values of the data (|log2FC|) > 1, and *P* < 0.05 is recognized as differential indication of genes [18]. Finally, in order to improve the appropriateness of differential expression genes, the FunRich soft device (text 3.1.3) was applied to obtain three numerical focusing genes that were all upregulated or downregulated, which was used to elaborate in the second step. The corresponding difference between selection and overall survival indicates a gene [19].

### 2.3. Differential Genes Were Selected

The digital gene expression demonstration tool was selected using the SAGE Genf database provided by CGAP. Select two pools of breast cancer tissue and benign breast tumors, and configure the *F* value to be 2; that is, the expression difference is more than 2 times; *Q* is 0.1. Differentially expressed genes are sorted by difference significance, strength, or weakness, and differential genes are evaluated in both short and long sequence tag libraries. Bioinformatics analysis was carried out on a highly expressed sequence FAM83A with unknown function [20].

### 2.4. Sequence Alignment

The EST database, nr database, and pro databases were retrieved using the BLAST software. Homology analysis of the copied gene nucleotide sequences with the nucleotide sequences already known in Gene Bank. Amino acid sequence similarity analysis was used with NCBI/BLAST and multisequence alignment and evolutionary tree analysis with Clustal W [21].

### 2.5. Physicochemical Properties and Subcellular Localization

Physical and chemical properties such as protein molecular weight, isoelectric point, and hydrophobicity were analyzed using ExPASy ProtParam. Subcellular localization was predicted using the PSORT II service program.

Signal lP is used for signal peptide and shear site prediction. Secondary structure and conservative domain prediction are predicted with SOPMA tools and NCBI/CDD, respectively [22].

### 2.6. Electron Expression Spectrum Analysis

FAM83A is obtained by analyzing EST expression in the UniGene library with FAM83A as the keyword gene electron expression profiling.

To illustrate the differential indication of the effect of the gene on the overall survival of breast cancer patients, in the Kaplan-Meier plotter numerical library (http://www.kmplot.com/), patient samples are divided into high expressive groups and low expressions according to the median indication of gene group [23]. Using tacit parameters, the median survival period of each gene in the high and low expression groups was calculated; if log rank *P* < 0.05, the gene was considered to indicate a difference with the overall survival period [24].

### 2.7. Illustrate the Differences Corresponding to the Overall Survival Period to Indicate the Efficacy of Genes

Gene Ontology (GO) enrichment and Kyoto Encyclopedia of Genes and Genome (KEGG) pathway enrichment analysis were used to identify the efficacy of genes. In this study, the application of the clusterProfiler package in the RStudio software device to the corresponding differences in the overall survival of breast cancer shows that the gene holds GO elaboration and KEGG elaboration; *P* < 0.05 is considered to have statistical significance (Figure 1) [25].

### 2.8. Protein-Proteins Mutually Select and Select Each Other's Functions

Network protein-protein functions play a crucial role for each other in adjusting biomimetic processes. The function of each other plays a crucial role in adjusting the biometric process. This type of relationship can pass the protein-protein interaction (PPI) network performance, each contact represents a protein, and the side represents the egg white matter with the function of each other. Tightly packed areas can be used as enrichment effect groups. The STRING Library (https://string-db.org/) contains a wealth of information about the functions of the egg white matter and each other. For the sake of evaluation and the corresponding differences in overall survival, the correlation between the causes is indicated in the difference indication gene list into the STRING value library. The specified reliability is 0.4; catch the PPI table data into the Cytoscape soft device to form a PPI network and apply the unplugged molecular synthesis test in the soft device (MCODE score > 4 points and the number of sections > 5) to select the pivot modules in the PPI network. Finally, pass the CytoHubba plug-in to calculate each in the network. The maximal clique centrality (MCC) score of a gene takes the top 10 genes as the central genes [26].

### 2.9. Pivotal Genetic Verification

Numerical Library Research Pivot New Gene Indication Using Database and Human Protein Atlas (HPA) were used for the verification of key protein. Examination of the indication of the mRNA and egg white grades of the central gene between breast cancer tumor tissue and normal tissue was performed [27].

## 3. Results

### 3.1. Highly Expressed Gene Selection in Breast Cancer

Finally, 33 genes that were highly expressed in breast cancer were selected. More than half of these were injected into the gene pool, from which a function cannot have high expression gene FAM83A which was extracted. The results of the Select Short Tag Sequence search show that 31 of the 38 short sequence tag libraries have FAM83A representative tags (ATGTACAGGT). Within the seven libraries of short sequence labels for benign breast tumors, two libraries have this representative label, with a difference in expression of 7.46-fold. And, within the 23 breast cancer long sequence label library, 20 have FAM83A stands for label (ATGTACAGGTTTGTAGC) and have appeared 964 times in total. And in the five benign breast tumor long sequence label libraries, only 1 library has this representation label; the expression difference is 3.14 times [28]. Upload a list of differentially expressed genes associated with overall survival to STRING, and set a reliability of 0.4 to determine whether the interaction is meaningful. The PPI network is constructed (Figure 2).

FAM83A sequence comparison results and different splicing body composition in Gene Bank using BLAST tool were evaluated, the result sequence is highly homologous to FAM83A, and most of them are human new mRNA sequence.

Hub genes are a class of genes that play a crucial role in biological processes. Genes and other nonhub genes in the related pathway are often regulated by this. Therefore, pivotal genes may become biomarkers and therapeutic targets for breast cancer. Using Cytoscape's plug-in CytoHubba, the top 10 hub genes were obtained by MCC method, which were NDC80, BUB1, CDCA8, FAM83A, BIRC5, CCNB1, KIF2C, CENPF, MAD2L1, and CDC20 (Figure 3).

Two of these sequences are transcriptional variants of FAM83 A, with Gene Bank login numbers NM-207006 1 and NM-032899. Comparing the similarities of various amino acid sequences of FAM83A, humans and gibbons, mice, turkeys, and clawed toads were 98%, 87%, and 64%, respectively; 41% of the amino acid composition is more robust in vertebrates.

To further understand the function of these genes, RStudio software used clusterProfiler package for the resulting lifetime-dependent differential expression.

For functional analysis of genes, *P* < 0.05 was considered statistically significant. GO functional analysis showed that the function of these genes was mainly related to cell division and related to biological processes (Figure 1). KEGG pathway analysis revealed these bases because of participating in cell cycle, human T cell leukemia virus 1 sense.

The sequence size of each species is similar, and the starting amino acid is methionine. Given the FAM83A multisequence comparison of evolutionary tree analyses, humans and gibbons are evolutionarily closer, and there are also relatively close evolutionary sources in other species (Figure 4) [29]. 10 hub genes were obtained by Oncomine database and HPA database pair screening. The expression of hub genes was verified. Oncomine database results show that BIRC5, CDC20, NDC80, CENPF, MAD2L1, CDCA8, and KIF2C and levels of BUB1, FAM83A, and BUB1B were significantly upregulated in breast cancer tissues (Figure 4). The above results suggest that the hub genes screened have good robustness.

Physicochemical properties and subcellular localization FAM83A (AF497803) consist of 367 amino acids, and the biological software predicts the relative molecular mass of 40606 and the isoelectric point of 8.97. The half-life of the egg's white matter in humans is 30 hours for reticulocytes; the instability index is 51.49 (above 40, considered unstable), the type is unstable protein, the fat index is 77.06, the average hydrophobic value is -0.346, and it is hydrophilic egg white matter. According to software analysis, the probability of predicting the expression of this protein in mitochondria is slightly greater (435%), followed by the nucleus (348%) and cytoplasm (217%), respectively [30].

Protein structure ELM prediction found that there are phosphorylation sites such as Pk and PKA, MAPK action recognition sites, SH2, SH3, RPEL, and WH2 combined with the motif, and no conservative domains were found. No signal peptide shear sites were predicted. The SOPMA method predicts the secondary structure, and the results show that the A-helix accounts for 43.5% of the FAM83A, *β* folding accounted for 5.72%, and extended chains and irregular curl structures accounted for 11.99% and 485%, respectively [31].

FAM83A gene expression electronic indication profiling is shown in Table 1. FaM83A gene is expressed in some normal tissues and a variety of tumors.

FAM83A is found in breast cancer cell lines and breast cancer tissues. The RT-PCR results showed that FAM83A was present in both breast cancer cell lines MDA-MB-231 and MCF-7 Da (Figure 2(a)). Of the 5 breast cancer tissues, 3 were highly expressed, and none was expressed in the responding paracancerous tissues and breast fibromas [32].

The gene and coding product sequence information of FAM83A was obtained from the Gene Bank database for the analysis of gene structure. Spidey was used to obtain the exon and intron information of the genes. To explain the coding product, we use the ExPASy (http://www.expasy.org) tool to expand the physicochemical analysis of egg white. Subcellular localization of proteins was premeasured using PSORT II. There is also NCBI's Conserved Danaiis that predicts the functional sites and structures of proteins; explore the possible functional orders of proteins; use the TM-HMM site to solve whether the protein encoded by this gene has a transmembrane structure. SignalP 3.0 server (http://www.cbs/dtu.dk/service/SignalP/) predicts that the protein has no lysis site with signal peptide. UniGene via NCBI (http://www.ncbi.ntn.nih.gov/entiez/<juery.fcgj.db=unigene), and SOURCE (http://genome—www5.The.slanfoid.edu/cgibin/souce/souceSeach) database looks at the gene in different tissues, growth stages, and relative expression of biological function pathological states. The protein homologous to the gene sequence was retrieved, and the Clustal X software was used to perform multisequence comparison of homologous proteins and construct a multispecies evolutionary tree, and the bootstrap method was used to generate random seed self-testing 1000 times to verify the reliability of the evolutionary tree, using MEGA 3 1 to observe the evolutionary tree results (Figure 5) [33].

57 differentially expressed genes were analyzed by DAVID website GO functional enrichment analysis and KEGG pathway enrichment analysis; GO analysis included biological processes (BP), cellular components (CC), and molecular function (MF). Biological processes include ureter germination and development. The downregulated genes were significantly enriched in lipid metabolism.

### 3.2. RT-PCR Verification Expression

In this test, 231, 435, MCF-7, HELA, A2780, and AN3CA cell lines were tested, all originated from xx tumor testing room. Following the NCBI GenBank FAM83A mRNA sequence, use Olgo6 0 to design the detection primers located inside the reading frame near the 3′end of the sequence. The upstream primers are 5′AAACAAAG-GCAGCAGTTCCACTC′3, and the downstream primers are 5′TCATGGCCAA-GAGACGCACAG′3; the primers were synthesized by Invitrogen, using the envisioned PCR product BLAST from the National Biotechnology Center's (NCBI) nucleic acid nonredundant database, and the specificity of the product is known to be excellent from the search results. The amplification was performed using dual-temperature PCR after predictive exploration, and the conditions are as follows: 95 degrees, 5-hour predeterminability, 94 degrees 30 s, 70 degrees 2ni, and 72C 10 mn after 34 cycles prolong. Amplification tubes use the gene G3PDH as an internal reference to test the reach of FAM83A in the tumor cell line described above, PCR. The product is cloned into the T vector and sequenced in the same sequence as the gene of interest [34].

The general term for FAM83A is family sequence with similarity 83, member A. Gene ID is 286077. Databases such as Gene Ontology and KEGG are uncommented and have no research reports on their structure and function. There is a valuable study of this gene. The newly submitted DNA of this gene is 5604 bp. The full length CDS zone is located between 70 and 3609 bp, encoding the full length 1179aa's hypothetical protein LOC286O77. GenBank's reference sequence is NP—940890. Spidev (http://www.ncbintmnihgov/EBResearch/Ostell/Spidey/) compared the sequence of mRNA parameters of FAM83A with the corresponding gene full length sequence. The gene was shown to have 5 exons and 4 introns (see Table 2). In this case, both sides of the four introns conform to the “GT-AG” shearing rule [35].

ExPASy's analysis software ProtParam predicted that the molecular weight of the gene-coded protein (NP-940890) would be 127101. 3Da theory isoelectric point pl = 6 61 ProtScale's Kyte and Doolittle method predicted the hydrophobicity of a protein, showing no significant hydrophobicity of the protein. PSORT H's K-NN method predicts that the probability of the protein being localized within the nucleus is 609% and the probability of locating the mitochondria is 26.1%, so it is likely to be an intranuclear protein (Figure 6) [36].

Using both InterProScan and MotifScan, it is predicted that there is 1 function at this protein (4-284). The domain DUF1669 (*E* = 0.00004) is unknown, which is 8 in the FAM83 protein family. Species of proteins are found except FAM83G; in proteins (94-288) aa, 1 phospholipase D/nuclease functional domain (*E* = 0.00006) is stored with the activity of phospholipase D and nucleic acid endonuclease, and PLD can hydrolyze the phosphodiester bonds of phospholipids, resulting in phospholipidic acid and 1 hydrophilic components such as choline; phosphatidic acid appears to be an important molecule involved in signal transduction. MP dehydrogenase/GMP reductase domain functional domain is found at (121-852) aa and many possible functional sites, such as ASN glycosylation site, AMP phosphorylation site, CK2 phosphorylation site, and PKC phosphorylation sites. Submit the sequence to SMART (http ://smart embl heidelbeig de/ amart/show motifs pl), ScanProsite (hp //www- expasy- ch/tools/ scan- prosite/), and ProClass (htp //pir geo ge town edu/piiwww/ seach/pattem shtml). The site also found the above implicit functional sites. ELM also found a multiple function basis: PLCXc functional domain (phospholipase C and catalytic domain X), which acts as a signal messenger in the signal transduction of eukaryotes and is in the protein of the (107-237) aa, and Prim Zn Ribbon functional domain and FYVE (protein present in Fab1 YOTB, Va1, and EEA1) functional domains, which are all joint sites of Zn ions [37].

TMHMM predicted that the protein encoded by this gene would not be able to display a transmembrane structure. The SignalIP30 attendant predicted that the protein does not have a lysis site for the signal peptide, indicating that the protein is most likely a nonsecretory protein. Follow the SOURCE and UniGene databases for the ESTEST sequence content of the gene to initially estimate the relative expression of the gene in normal and tumor tissue. The gene is most expressed in normal tissues in SOURCE in the front glands and cervix [in tumor tissues = 1112/1192(93%), positives = 1123/1192(94%)] using chstak for multisequence comparison and the results of the species evolutionary tree [38]. This is shown in Figure 6.

From 1 to 6, it is 231,435s, MCF-7, heb, A2780, and AN3 CA. The PCR product of FAM83A in the cell line is about 200 bp in size, which is equivalent to the actual size of 182 bp.

RT-PCR product results were detected by 20% agarose gel electrophoresis to see specific amplification bands in each tumor cell line, and their molecular weight size was consistent with the expected results (Figure 1). 231, 435s, MCF-7 heh and ovarian cancer A2780 cell line and endometrial cancer AN3 CA. The FAM83A in the cell line is expressed, and the PCR product delivery sequence is consistent with the actual gene sequence of interest [39].

A is expressed in breast cancer cell lines, a is MDA-MB-231, and b is MCF-7; B is at 5 manifestations in cases of breast fibromas; C in 5 cases of breast cancer and their paracancerous tissues; and 1, 3, 5, 7, and 9 lines for breast cancer tissue; 2, 4, 6, 8, and 10 lanes are the corresponding paracancerous tissues.

## 4. Discussion

The mammary gland is the organ that most often develops benign and malignant tumors, and cancerous hyperplasia is fundamentally different from benign tumors, and the treatment plan is completely different. Therefore, when selecting high expression genes for breast cancer, clinicians hope to look for genes that are highly expressed in cancer tissues and are not expressed or low expression in benign tumor tissues, which are more valuable for helping clinical diagnosis and treatment [40]. The CGAP SAGE database can analyze tumor tissue gene expression profiles and look for tumor-specific expression of new genes in the SAGE library. Two pools of breast cancer and benign breast tumors were selected, and the library of benign breast tumor pools was found in 7 short sequence labels and 5 long sequence labels, mainly breast fibroma, breast muscle epitheliomas, and benign mammary stromal tumors, and breast cancer high expression gene FAM83A was selected. Furthermore, the semiquantitative RT-PCR results further confirm the reliability of bioinformatics databases. This gene is highly expressed in breast cancer cell lines and in several breast cancer tissues [41].

At present, FAM83A has been studied very little, and only the gene is used as a tumor biological marker for the detection of peripheral blood, but the function of this gene is rarely reported. ELM analysis revealed that the protein has LIG_14-3-3_1 and LIG_ 14-3-3_3 protein ligands, and cyclin substrates identify sites and PK PKA phosphorylation sites, etc. 14-3-3 proteins are a family of conserved proteins in eukaryotes, which play a role in cell transduction, cell cycle regulation, apoptosis and stress response, and tumor malignant transformation, and are the mediators and regulators of the interaction between proteins. C10\Cyclin substrate identification sites are found in cyclin/CDK interaction proteins [42]. The presence of this motif in the CDK increases the phosphorylation level of the (ST) Px (KR) motif. It is identified by conserved regions in the cyclin protein and binds to a p21Kip cyclin-like method. PK and PKA phosphorylation sites are common molecular structures in signaling regulation and have a wide range of regulatory roles in cell proliferation and cell cycles [43].

The above analysis found that the protein is evolutionarily robust, from low to high animals having similar protein expression, is an unstable hydrophilic protein, may be localized on the mitochondria, and has multiple functional sites and motifs, indicating participation in signal transduction and cell cycle regulation. It is important to mention that there are multiple transcriptional variants, indicating that they play an important role in the regulation of cell proliferation and apoptosis during the development of organisms. The high expression of this gene in breast cancer has obvious significance, most likely by making cells continue to proliferate, control apoptosis, and change the cell cycle [44].

FAM83A is a gene expression material available in SAG's DGED database and bioinformatics analysis. The corresponding unknown functional genes associated with breast cancer are rarely explained, and there are no reference materials, and it is difficult to study them by traditional methods. We use a variety of bioinformatics resources and tools to analyze and obtain a lot of meaningful information [45].

InterProScan predicted that the gene encodes the protein‘s (4-284) aa with an unknown function of 1 domain DUF1669, 55 proteins from high-level animals such as humans and mice to low-grade zebrafish and African claw frogs. The detailed function of the functional domain is unknown, but it can be seen that it is very conservative in evolution. Prediction shows the presence of 1 functional domain with phospholipase D/nuclease at (94-288) aa of the protein. The nuclease superfamily has a common motif HxK (x)4D (x)6GSxN with signal transduction, lipid biosynthesis, pathogenic bacteria, and viral restriction nucleic acid endonucleases related to signaling that affect ejection and cell drink and receptors [46] and regulation of actin cytoskeletal reorganization. Intercellular membrane transport is controlled, while it itself is controlled by phosphatidylinositol 4,5-diphosphate, PKC ADP-related factor, and rho family GTPase tuning. In contrast to these two functional domains, their positions on proteins overlap and intersect, which is explained in InterProScan [47]. The department members of the DUF1669 family have recessive phospholipase activity, so it can be inferred that the function of the DUF1669 functional domain is likely to be similar to that of phospholipase D/nuclease. Functional domains are similar and play an important role in signal transduction of tumor cells, among other things. MotifScan predicted that the gene has multiple phosphorylation sites, binding PSORT H to its subcellular localization in the nucleus. It can be speculated that the gene can not only play a role in regulating signal transduction but also be adjusted by other adjustment proteins and has a number of adjusted functional sites, such as phosphorylation sites. ELM predicts that it has a PLCXc domain of phosphoyositol-specific phospholipase C, with MotifScan [48]. Predicted results with phospholipase D functional domains are similar. In addition, ELM predicts many functional orders, such as ST1 functional domains, Prim Zn Ribbon, and FYVE functional domains, which suggest that the gene is roughly as close as it is within the nucleus small molecules or Zn ions bind to function. Using Clustal X to carry out multisequence comparison and composition to construct each species, it can be seen in the evolution tree that the gene expression product is homologous to the proteins of multiple species, and the results of multi-sequence comparison are shown. The gene encodes proteins with very conservative amino acid sequences, which are probably related to their structure and function [49]. After RT-PCR testing, the product of FAM83A was detected by agarose gel electrophoresis to detect 1 specific amplified band, and its molecular weight size was consistent with the expected results, which verified the group. It is indeed expressed in breast cancer and several other tumor cell lines. Future work will collect normal breast tissue and breast cancer specimens, take fluorescence quantitative PCR and other methods to detect the relative expression of the gene in breast cancer and normal tissues, and design a well-thought-out experiment to explore the structure and function of the gene in depth [50].

## 5. Conclusion

FAM83A is a potential research target associated with tumorigenesis and metastasis. Initial tests confirmed the expression of this gene. To lay a solid foundation for further learning. FAM83A is a highly expressed gene in breast cancer and can serve as a target for studying molecular mechanisms in breast cancer.

## Figures and Tables

**Figure 1:** GO function analysis and KEGG pathway analysis of differentially expressed genes associated with overall survival. KEGG pathway analysis revealed these bases because of participating in cell cycle, human T cell leukemia virus 1 sense.

**Figure 2:** PPI networks of differentially expressed genes associated with overall survival. Upload a list of differentially expressed genes associated with overall survival to STRING, and set a reliability of 0.4 to determine whether the interaction is meaningful. The PPI network is constructed.

**Figure 3:** 10 hub genes and their interactions were obtained by MCC method. The top 10 hub genes were obtained by MCC method, which were NDC80, BUB1, CDCA8, FAM83A, BIRC5, CCNB1, KIF2C, CENPF, MAD2L1, and CDC20.

**Figure 4:** The transcriptional level of hub genes was verified by Oncomine database. Oncomine database results show that BIRC5, CDC20, NDC80, CENPF, MAD2L1, CDCA8, and KIF2C and levels of BUB1, FAM83A, and BUB1B were significantly upregulated in breast cancer tissues.

**Figure 5:** GO enrichment analysis of differentially expressed genes ((a) upregulated genes and (b) downregulated gene; *P* < 0.05).

**Figure 6:** Kaplan-Meier prognostic value of core genes (log rank *P* < 0.05 considered statistically significant).

**Table 1:** FAM83A gene electron indications.

Organization	Transcript/million	Organization	Transcript/million
Mouth	1 476	Head/neck cancer	792
Larynx	414	Lung cancer	203
Neck	103	Bladder cancer	171
Esophagus	98	Prostate cancer	136
Prostate	89	Pancreatic cancer	57
Lungs	74	Esophageal tumors	57
Bladder	67	Leukemia	52
Marrow	61	Breast cancer	51

**Table 2:** Exon and intron layout prediction for FAM83H.

	Genomic coordinates	mRNA coordinates	Length	Identity mismatches		Gaps	Donor site	Acc. site
Exon 1	1-54	1-54	54	100.0%	0	0	d	
Exon 2	3148-3609	55-516	462	100.0%	0	0	d	a
Exon 3	44224586	517-681	165	99.4%	1	0	d	a
Exon 4	4654-4778	682-806	125	100.0%	0	0	d	a
Exon 5	5022-9812	807-5587	4781	99.7%	14	10		a

## Data Availability

The data used to support this study is available from the corresponding author upon request.
